# An Improved Strategy for Task Scheduling in the Parallel Computational Alignment of Multiple Sequences

This article has been retracted.

**DOI:** 10.1155/2022/8691646

**Published:** 2022-01-28

**Authors:** Muhammad Ishaq, Asfandyar Khan, Mazliham Mohd Su'ud, Muhammad Mansoor Alam, Javed Iqbal Bangash, Abdullah Khan

**Affiliations:** ^1^Department of Computer Science and IT, Agriculture University Peshawar, Pakistan; ^2^Faculty of Computing and Informatics Multimedia University Malaysia, Malaysia; ^3^Faculty of Computing, Riphah International University, Islamabad, Pakistan

## Abstract

Task scheduling in parallel multiple sequence alignment (MSA) through improved dynamic programming optimization speeds up alignment processing. The increased importance of multiple matching sequences also needs the utilization of parallel processor systems. This dynamic algorithm proposes improved task scheduling in case of parallel MSA. Specifically, the alignment of several tertiary structured proteins is computationally complex than simple word-based MSA. Parallel task processing is computationally more efficient for protein-structured based superposition. The basic condition for the application of dynamic programming is also fulfilled, because the task scheduling problem has multiple possible solutions or options. Search space reduction for speedy processing of this algorithm is carried out through greedy strategy. Performance in terms of better results is ensured through computationally expensive recursive and iterative greedy approaches. Any optimal scheduling schemes show better performance in heterogeneous resources using CPU or GPU.

## 1. Introduction

This research paper proposes a novel dynamic programming-based task scheduling for parallel multiple sequence alignment (MSA). Further modifications in the proposed algorithms, like iterative, recursive, and greedy strategies, enhance the performance of scheduling in any parallel system. The application of dynamic programming optimization for task scheduling in case of parallelized multiple sequence alignment is preferred over other dynamic task scheduling approaches.

The complex issue of task scheduling in any parallel processor system has multiple possible solutions. The structure of a problem like task scheduling can be characterized, then, the application of dynamic programming is the best solution. Multiple alignment operation is divided into pairwise alignments or subparts. Pairwise alignments are interrelated, and the solution of one section can be used in another part of the same problem. The same problems here mean the complete multiple alignment. In this recursion, the intermediate results are stored in a matrix where they can be recalled later in the same program.

The storage of profile alignment or intermediate results is different in each individual computational multiple sequence alignment. In dynamic programming, the structure of an optimal solution is characterized, then, the value of an optimal solution is defined recursively, and then an optimal solution is constructed from the computed information. In any array of parallel workers, a master node collects the profile scores. Similarity of sequences is determined from the alignment score or computed information. In dynamic algorithm, the exponential cost is reduced to polynomial type, so more efficient than the ordinary divide and conquer algorithm in terms of time complexity. Dynamic programming application for any stated problem is diagrammatically shown in Figure 1.

Homology modelling or potential orthologues and paralog description is also possible on the basis of protein structure comparison [1].

In a given protein structure, if the amino acid shows the interaction or association with other subunits and different atoms, then, it is called as quaternary protein structure.

Primary structure of proteins as visible in Jalview with PDB ID 4HHB. This structure is retrieved from Protein Data Bank (PDB). The primary structure is shown in Figure 2. The figure shows sample word-based sequences. Three dimensional protein structure matching is more accurate and comprehensive in terms of structure and function prediction but requires a lot of processing time.

There are many need-based word-based sequence alignment visualization tools.  Figure 3 is the visualization of sample dataset. In Bioinformatics, the notion of tertiary structure is usually used for proteins rather than nucleic acids.

Greedy approach improves the efficiency of the dynamic algorithm by reducing the local maxima or the number of possible choices. Computationally complex recursive and iterative greedy techniques further enhance the application of this hybrid methodology.

## 2. Related Research Work in Parallel Processing of MSA

Remote homologue proteins improve sequence alignment by retrieving structural specifications from multiple structure alignment profiles. Sequences that share the same ancestry are called as homologs, and there are two kinds of homologs, orthologs and paralogs. In one approach, the score functions were combined with a systematic search algorithm. The score functions were based upon the sequence and structural information [2]. Sleater et al. proposed the MSA algorithm to be run in a parallelized fashion with the sequencing data distributed over a computer cluster or cloud-based server farm. The cloud computing technology improves the speed, quality, and capability of MSA. They introduce the next generation of cloud-based MSA algorithm [3]. Some researchers utilize BlueGene/Q or JUQUEEN supercomputing capability to evaluate the performance of parallel multiple sequence alignment. A parallel I/O interface for simultaneous and independent access to a single files collectively has been designed and verified [4]. Diaz and his coresearchers developed MC64-ClustalWP2 as a new implementation of ClustalW algorithm. They integrate a novel parallelized strategy that significantly increases the performance of alignment. The proposed method is useful when aligning long global sequences by using multicore architecture or with many processor cores [5]. Their hardware and software feature analysis were carried out for the exploitation and optimization of full potential in case of a parallelized system. To test the performance of their proposed algorithm, they use a hybrid computing system. The researchers counted manifold benefits of MC64-Clustal WP2 [6]. To improve the scalability of global sequence alignment, an MPI-based parallelization technique is proposed. In this method, a parallel waveform algorithm based on a chunk size transformation to handle large datasets with message passing model exposes high speed up and scales linearly with the increasing number of processes [7]. Some researchers examine different multicore machines by running a variety of MSA software [8]. In recent years, we observe various kinds of novel techniques for parallel MSA like artificial bee colony optimization [9]. R is extensively used for computational sequence alignment [10].

## 3. Problem Statement regarding Multiprocessor Task Scheduling through Dynamic Programming

In parallel MSA, we deal with the multiprocessor scheduling system. Assume that a set of tasks is to be executed by a parallel system with identical processors. For example, task *Xi* requires time *Ti* for execution.

Task here means a single pairwise word-based or structure-based alignment. In this case, the precedence of task execution is achieved by a tree or forest of tree data structure. Dynamic programming like genetic algorithm takes in to account all possible candidate solutions, which is not an efficient approach.  Figure 4 shows the parallel processing of MSA, and each worker is responsible for one PWA at a time.

## 4. Application of Dynamic Programming for Task Scheduling Problem in MSA

In case of sequential or parallel processing of each pairwise alignment in MSA, a single task (pairwise alignment) is selected by each processor. Thus, an algorithm based upon dynamic programming can solve the task selection problem. If we have a set *S* = {*x*_1_, *x*_2_, *x*_3_ ⋯ .*x*_*n*_} of *n* tasks. Each pairwise alignment (*x*_*i*_) has a starting time *S*_*i*_ and a finishing time *F*_*i*_ where 0 ≤ *S*_*i*_ < *F*_*i*_ < ∝. The tasks are sorted with respect to increasing finish time *F*_1_ < *F*_2_ < *F*_*n*_. For scheduling tasks during MSA, the profile makes require the maximum size subset of closely related sequences. The aligned sequences make a profile. Pairwise alignments (tasks) cannot use a given processor at a time. Each task has a corresponding time interval *T*_*j*_ = *S*_*j*_, *F*_*j*_ during which the processor is busy in executing the task. For a given two tasks *x*_*i*_ and *x*_*j*_, the interval *T*_*i*_ and *T*_*j*_ do not overlap, i.e., *S*_*i*_ ≥ *F*_*j*_or*S*_*j*_ < *F*_*i*_. So all tasks for a given processor must be compatible in terms of their ordered time interval.

If *X*_*ij*_ is the set of all tasks *a*_*k*_ in *X* which is started when *a*_*i*_ finishes and finish before task *a*_*j*_ starts. *X*_*ij*_ = {*a*_*k*_∀ *X* : *F*_*i*_ ≤ *S*_*k*_ < *F*_*k*_ ≤ *S*_*j*_} here *F*_*i*_and *F*_*k*_ denote finish time of *a*_*i*_ and *a*_*k*_.

*S*_*k*_and *S*_*j*_ represent start time of tasks *a*_*k*_ and *a*_*j*_. If *i* = 1 and *j* = *n* then *X*_*ij*_ exclude task *a*_1_ and *a*_*n*_.

For this purpose, we can define fictitious tasks *a*_0_and *a*_*n*+1_ such that the finish time of *a*_0_ is *f*_0_ = 0 and the start time of *a*_*n*+1_ is *S*_*n*+1_ = ∝. So 0 ≤ *i*, *j* ≤ *n* + 1 and *X*_0 *n*+1_ include all tasks including *a*_1_ and *a*_*n*_.

Based upon *a*_*k*_ task *X*_*ij*_ can be divided into *X*_*ik*_ and *X*_*kj*_. All *X*_*ik*_ tasks start after *a*_*i*_ finishes and finish execution before *a*_*k*_ starts execution. Similarly, all *X*_*kj*_  tasks start execution after *a*_*k*_ finishes and finish before *a*_*j*_ starts. *X*_*ik*_ and *X*_*kj*_ are subsets of *X*_*ij*_, but *X*_*ij*_ ≠ *X*_*ik*_ ∪ *X*_*kj*_ or *X*_*ij*_ = *X*_*ik*_ ∪ *X*_*kj*_ ∪ *a*_*k*_ because *a*_*k*_ does not exist in both subsets.

A sample parallel web-based reference tree generation of 38 RefSeq Proteins is shown in Figure 5.

Also, the solution of *X*_*ij*_ can also be demonstrated as

(1) $$\begin{array}{c} Sol\left(X_{ij}\right)=Sol\left(X_{ik}\right)\cup Sol\left(X_{kj}\right)\cup \left(a_{k}\right). \end{array}$$

If *Sol*(*X*_*ij*_) is an optimal multiple sequence alignment, then, *Sol*(*X*_*ik*_) and *Sol*(*X*_*kj*_) are also optimal. If we have another solution *Sol*(*X*_*ik*_)′ for *X*_*ik*_, and we replace *Sol*(*X*_*ik*_) in *Sol*(*X*_*ij*_) with *Sol*(*X*_*ik*_)′ then *Sol*(*X*_*ij*_)′ has more tasks than  *Sol*(*X*_*ij*_).So  *Sol*(*X*_*ij*_) is not optimal, and we encounter a contradiction so it is proved that *Sol*(*X*_*ik*_) and *Sol*(*X*_*kj*_) are also optimal set of tasks.

## 5. Recursive Solution of the above Strategy

Recursion is computationally expensive. Assume that *L*[*i*, *j*] is the number of tasks in a maximum size subset of mutually compatible tasks in *X*_*ij*_. If *X*_*ij*_ = ∅; then, *L*[*i*, *j*] = 0. We know that *Sol*(*X*_*ij*_) = *Sol*(*X*_*ik*_) ∪ *Sol*(*X*_*kj*_) ∪ (*a*_*k*_) so the recurrence relation for the problem is *L*[*i*, *j*] = *L*[*i*, *k*] + *L*[*k*, *j*] + 1. The recursive definition of *L*[*i*, *j*] becomes

(2) $$\begin{array}{c} L\left[i,j\right]=\left\{\begin{array}{cc} 0, & \text{if }X_{ij}=\emptyset ,\\ \max\text{of}\left\{L\left[i,k\right]+L\left[k,j\right]+1\right\}, & \text{if }X_{ij}\neq \emptyset ,\\ i<k<j. \end{array}\right. \end{array}$$

There is no restriction of using sequence data sets. Sequences of any specific organism are not mandatory.  Figure 6 shows the chloroplast protein sequences, and chloroplast is a green pigment in many plants, responsible for photosynthesis.

## 6. Greedy Approach and Its Implications for the Abovementioned Problem

Greedy approach increases the efficiency of the algorithm by reducing the search space and reduces the computational complexity. If we have nonempty subproblem *Y*_*ij*_ and *c*_*m*_ is any task in *Y*_*ij*_ with earliest finishing time. The optimal task or the task with the earliest finishing time (quick execution) is called *c*_*m*_.

The following steps should be proved for the application of greedy solution in the abovementioned task scheduling algorithm. Greedy strategy takes into account the most optimal sequences to be aligned with a given MSA profile.

In the first step, the determination of the suboptimal structure of the problem is carried out. We have to prove that the task *c*_*m*_ can be used in some maximum size subset of mutually compatible tasks of *Y*_*ij*_. And the subproblem *Y*_*im*_ is empty, so that choosing *c*_*m*_ leaves the subproblem *Y*_*mj*_ as the only one that may be nonempty.

First of all, we have to prove the second simple problem that *Y*_*im*_ is empty. Lets *Y*_*im*_ is nonempty, it means that there is some task *a*_*k*_ such that *f*_*i*_ ≤ *S*_*k*_ < *f*_*k*_ ≤ *s*_*m*_ < *f*_*m*_⟹*f*_*k*_ < *f*_*m*_. So *a*_*k*_ is also in *Y*_*ij*_ but its finishing time is less than *c*_*m*_ which contradicts with our assumption that *c*_*m*_ has the earliest finishing time. We show that there is another task in *Y*_*ij*_ that has less finishing time than *c*_*m*_, and it proves that *Y*_*im*_ is empty.

In any approach, the power of computational techniques in case of translation as shown in Figure 7 cannot be ignored.

For a greedy approach to be applied in this case, we have also to prove that *c*_*m*_ can be used in some maximum size subset of mutually compatible tasks of *Y*_*ij*_ or *c*_*m*_ is a member of one of the optimal solutions. Suppose that *A*_*ij*_ is a maximum size subset of mutually compatible tasks of *Y*_*ij*_. Order *A*_*ij*_ is the monotonic increasing order of finishing time. Let *a*_*k*_ be the first activity in *A*_*ij*_ with respect to the finishing time. If *a*_*k*_ = *c*_*m*_ then we already know that and prove it before that *c*_*m*_ is used in some maximal subset of mutually compatible tasks of *Y*_*ij*_. Therefore, there is nothing to prove, and we show it that there must exist at least one of the optimal solutions which contain the task *c*_*m*_. So *c*_*m*_ belongs to  *A*_*ij*_ optimal solution.

If *a*_*k*_ ≠ *c*_*m*_; then, there must be some other optimal solution where task *c*_*m*_ exists. Lets suppose  *A*_*ij*_′ is another optimal solution and  *A*_*ij*_′ = *A*_*ij*_\{*a*_*k*_} ∪ {*c*_*m*_}.  *A*_*ij*_ tasks are disjoint, and it is true for  *A*_*ij*_′. This statement means that *c*_*m*_ belongs to  *A*_*ij*_′ because we negate *c*_*m*_ from  *A*_*ij*_′. As *a*_*k*_ is the first task in  *A*_*ij*_ to finish and the finishing time of *a*_*k*_ is greater than the finishing time of *c*_*m*_*f*_*m*_ ≤ *f*_*k*_. Here, *f*_*m*_ or *f*_*k*_ denotes finishing time of *a*_*k*_ or *c*_*m*_. So it means that task *c*_*m*_ is included in optimal solution set  *A*_*ij*_′ and  *A*_*ij*_′ is the maximal subset of mutually compatible tasks of *Y*_*ij*_. The number of tasks in  *A*_*ij*_ and  *A*_*ij*_′ is the same, and both have the same cardinality. We have proved that  *A*_*ij*_′ is a maximal set of mutually compatible tasks. All tasks in  *A*_*ij*_′ must be mutually compatible.

The conclusion of the above greedy approach is that task *c*_*m*_ belongs to *Y*_*mj*_ and *Y*_*im*_ = ∅. Therefore, it improves the efficiency of greedy approach in case of multitask scheduling algorithm compared to dynamic programming. In dynamic programming, there were two subproblems which were reduced to one by the greedy approach. The number of choices is *j* − *i* − 1 in dynamic programming, and there is only one choice in the greedy theorem.

Greedy algorithms do not work in some cases, i.e., in the cases of longest monotonically increasing subsequences. Suppose that we have a given sequence of <2, 3, 4, 13, 5, 6, 7>, and its longest common subsequence (LCS) is <2, 3, 4, 5, 6, 7>. If we solve this problem with greedy approach then its LCS is <2, 3, 4, 13> which is suboptimal. In greedy approach, the rest of three elements 13 cannot be chosen. Therefore <2, 3, 4, 13> is a monotonically increasing sequence, but it is not the longest monotonically increasing sequence. Figure 5 shows the export ability of candidate local optimal (sequences).

## 7. Structure of Recursive Greedy Algorithm for Task Scheduling

At each processor, the algorithm for task scheduling can be defined recursively. Recursive task selector (*s*, *f*, *i*.*j*) where *s* is the set of tasks and *f* is the finishing time. The initial value of *i* = 0 and *j* = *n* + 1. We want to determine a task that belongs to the optimal solution. In the process of recursion, there will always be an optimal or greedy choice.

Recursive task selector(*s*, *f*, *i*.*j*.).

Some computational alignment tools have unique ability to show translated proteins of given set of nucleic acid sequences as shown in Figure 8. Correct similarity index calculation of a given pairwise or multiple sequence alignment is principally related with gap and gap extension penalty as shown in Figure 9.

## 8. Structure of Iterative Greedy Algorithms for Task Scheduling in Parallel MSA

Iterative algorithms are more efficient than recursive algorithms. Recursive algorithms are computationally more expensive. The above recursive greedy algorithm can be expressed in an iterative manner. In task scheduling, we repeat the same process again and again, so iteration of the same process is computationally efficient. In this case, we have two tasks, *s* is set of all the tasks, and *f* is the set of the finishing time of all tasks.

Iterative task selector (*s*, *f*).

return *Sol*(*s*) //The set of all tasks that are mutually compatible is retrieved. Irrespective of whether recursive, iterative or any other hybrid modification to this approach, gap penalties of PWA or MSA are also essential as shown in Figure 7.

## 9. Implementation Details and Results

Multiple sequence alignment is a tightly coupled processing task, so the application of map-reduce model is not valid in the parallelization of MSA. The task scheduling during parallelization of MSA is based upon a single program and multiple data (SPMD) style. Imagine that the mesh cluster as discussed above is a global matrix of *m*∗*n* dimensions, and individual processors own a different collection of rows in the matrix. In this case, all processors are local, so each dimension receives a general block distribution object. Figures 8 and 9 can explain the strategy.

MPI I/O over a subset of MPI cores can also be used to foster file reading in any parallel MSA data set [11].

Figure 10 shows the famous machine learning approach for estimated diversion time calculation. The proposed scheduling algorithm using dynamic programming has O (nlogn) complexity. Each task or pairwise alignment (PWA) in the profile formation has a start and finish time. During the scheduling of MSA with multiple workers (processors), the goal is to overcome the overlap of any task (PWA) in any subset of the cluster mesh. The algorithm will also calculate the overall multiple alignment score.

In Python as a first step, a class task defines the start finish time with the calculated alignment score of each PWA. An iterative binary search is carried out to find the midpoint of any defined task with low and high indexes.

Substitution matrices are available in many libraries.

A variety of gap penalties can be opted. Some of the gap penalty functions available in Pymsa and other prominent matching libraries are as under.

Figure 11 is the conceptual design of mesh topology for parallel processing system. Some schedulers like the in-process use periodic jobs that use the builder pattern for configuration. These schedulers let you run the respective Python library functions periodically. The periodic time intervals are predetermined using a simple, human-friendly syntax.

In any parallel processing system, the following libraries need to be imported for task scheduling in your work space. These libraries include collections, datetime, functions, logging, random, re, and time.

Using Python object-oriented paradigm capability, the ScheduledTask in this case has eight user-defined functions for different operations. The job class has the default scheduler. Typical operations in process scheduling are time interval definition, excuse or run operation, clear cancel job, and the definition of next run. The scheduler also manages free time.

The main features of any scheduler should be (but not limited to) an efficient and effective execution of operations. It means fail load distribution and reduction in time complexity. There are simple to use API for scheduling jobs for simulated and real test bids. These API are very lightweight having no external dependencies, excellent test coverage, and tested on all latest Python 3 versions.

Tasks are scheduled based upon their finish time. As a convention of dynamic programming, the solutions of subproblems are stored in a matrix. The matrix stores the score of PWA or task till all elements in the array. The store results are used again and again in the profile building process of MSA. The entries in the matrix are filled recursively. At each step of parallel MSA, the alignment score is stored in a matrix. Large alignment scores replace the previous low scoring matrix.  Table 1 is only for three chloroplast protein sequences that can be extended to other species. Beside unique differences, the table shows identical and divergent sites.

In the first experiment, four tasks or workers get values. The time complexities remain less than many available optimal dynamic methods for this purpose.

Maximum likelihood estimate of Gamma parameter for site rates in case of protein sequences. The estimated value of the shape parameter for the discrete Gamma distribution is 0.5435.

Substitution pattern and rates were estimated under the Jones-Taylor-Thornton (1992) model (+G) [2]. A discrete Gamma distribution was used to model evolutionary differences among sites (5 categories, [+*G*]). Mean evolutionary rates in these categories were 0.03, 0.18, 0.50, 1.13, and 3.16 substitutions per site.

The amino acid frequencies are 7.69% (A), 5.11% (R), 4.25% (N), 5.13% (D), 2.03% (C), 4.11% (Q), 6.18% (E), 7.47% (G), 2.30% (H), 5.26% (I), 9.11% (L), 5.95% (K), 2.34% (M), 4.05% (F), 5.05% (P), 6.82% (S), 5.85% (T), 1.43% (W), 3.23% (Y), and 6.64% (V). For estimating ML values, a tree topology was automatically computed. The maximum Log likelihood for this computation was -119906.071. This analysis involved 10 amino acid sequences.

The number of amino acid substitutions per site from mean diversity calculations for the entire population is shown below. Analyses were conducted using the Poisson correction model. This analysis involved 2 amino acid sequences of the original chloroplast proteins. All ambiguous positions were removed for each sequence pair (pairwise deletion option). There were a total of 11039 positions in the final dataset.

Pseudomonas keratins multiple sequence alignment is shown in Figure 12. Optimal regions matching in any MSA depict the quality of algorithm.

Disorder comparison at each node of individual pairwise alignment is shown in Figure 13.

## 10. Discussion

Three dimensional comparisons of biological sequences involve the calculation of root mean square deviation, and parallelization of multiple protein 3D structure alignment reduces computational. This paper concludes a new technique for parallel MSA task scheduling using dynamic programming optimization in heterogeneous environments.

There are multiple choices during the scheduling of sequence matching tasks, so the application of dynamic programming (DP) is justified. DP is also used as a base method for computational sequence alignment. To further reduce the computational cost and to limit the number of candidate solutions, a greedy strategy is applied. Greedy approach does not take into account all candidate solutions in a single run.

Recursion and iteration solve the issue of optimal alignment score, but computationally expensive. In the era of fast processing machines, the greedy technique is not an efficient selection. Iteration is an efficient approach for optimal alignment and fair load distribution during parallel MSA task scheduling.

## Figures and Tables

**Figure 1:** Diagrammatic illustration of the conditions for the application of dynamic programming optimization.

**Figure 2:** Primary structure of human deoxyhemoglobin (4HHB, PDB ID).

**Figure 3:** Dataset from GenBank: the linear nucleotide chain constitutes the primary structure of nucleic acid. Here, nucleotides are represented by their respective word-based symbols.

**Figure 4:** Parallel processing of multiple sequence alignment.

**Figure 5:** Sample parallel tree generation using estimated Gamma parameters for local aligned site rates.

**Figure 6:** Chloroplast protein sequences of the given plant species.

**Figure 7:** Other sequence data export formats available in the majority of web-based implementation tools.

**Figure 8:** MSA of DNA sequences and the relevant translated proteins.

**Figure 9:** Pairwise and multiple alignment gap and gap extension penalty features.

**Figure 10:** Estimated diversion time calculation for parallel nucleic acid and protein computational sequence alignment.

**Figure 11:** Mesh type topology in case of cluster for protein structure MSA. One node in each row is a master node [12].

**Figure 12:** Graph showing results of six selected (NCBI GenBank) keratins (proteins) for MSA (word based).

**Figure 13:** Graphs show pairwise aligned protein sequences from each node in parallel system with disorder comparison at the middle of image.

**Code 1:** 

**Code 2:** 

**Code 3:** 

**Code 4:** 

**Code 5:** 

**Table 1:** Similarity parameters in the computational alignment of three chloroplast protein sequences.

Results from the Tajima's test for 3 sequences	
Configuration	Count
Identical sites in all three sequences	6261
Divergent sites in all three sequences	1284
Unique differences in sequence A	1043
Unique differences in sequence B	1282
Unique differences in sequence C	603

## Data Availability

The data used to support the findings of this study are included within the article. Computational MSA for the application of parallel system can be found [https://github.com/ishaqafridi/pyMSA.git]
